The article "Plasma miR-208b and miR-499: Potential Biomarkers for Severity of Coronary Artery Disease" was published in 2019. Journal: Dis Markers.

# Plasma miR-208b and miR-499: Potential Biomarkers for Severity of Coronary Artery Disease

**DOI:** 10.1155/2019/9842427

**Published:** 2019-11-22

**Authors:** Wei Wang, Tai Li, Lei Gao, Yang Li, Ying Sun, Heng-Chen Yao

**Affiliations:** ^1^Department of Cardiology, Liaocheng People's Hospital Affiliated to Shandong University and Clinical School of Shandong First Medical University, Liaocheng 252000, China; ^2^Department of Nursing, Liaocheng Vocational and Technical College, Liaocheng 252000, China; ^3^Zhong Yuan Academy of Biological Medicine, Liaocheng People's Hospital, Shandong University, Liaocheng, China

## Abstract

**Aims:**

MicroRNAs (miRNAs) are associated with the pathogenesis of coronary artery disease (CAD). The objective of this study is to explore plasma levels of miR-208b and miR-499 in CAD and analyze its association with the severity of CAD.

**Materials and Methods:**

195 consecutive CAD patients who underwent coronary angiography were enrolled in this study. Severity of coronary lesions was evaluated by the synergy between percutaneous coronary intervention with taxus and cardiac surgery score (SYNTAX) score (SS). Plasma levels of miR-208b and miR-499 were assessed by quantitative real-time polymerase chain reaction (qRT-PCR). The relationship between miR-208b and miR-499 and SS was analyzed.

**Results:**

The qRT-PCR results showed that plasma levels of miR-208b and miR-499 in SS > 32 (high SS) group was higher than those in low (SS ≤ 22) and intermediate (22 < SS ≤ 32) groups. Meanwhile, plasma miR-208b and miR-499 levels were significantly positive correlated with the SS (Spearman's *r* = 0.535 and *r* = 0.407, respectively; both *p* < 0.001). Multivariate logistic analysis results showed that miR-208b (odds ratio [OR]: 2.069; 95% confidence interval [CI]: 1.351-3.167; *p* = 0.001) and miR-499 (OR: 1.652; 95% CI: 1.222-2.233; *p* = 0.001) were independent predictors of high SS. In receiver operating characteristic curve, the area under the curve of miR-208b and miR-499 in prediction of high SS was 0.775 and 0.713, respectively.

**Conclusions:**

Higher plasma levels of miR-208b and miR-499 were positively associated with the severity of CAD, and plasma miR-208b and miR-499 can act as potential biomarkers for estimating the severity of CAD.

## 1. Introduction

Coronary artery disease (CAD) and its clinical complications is still a major cause of death in the world [1, 2]. The severity of CAD is closely associated with mortality, and the synergy between percutaneous coronary intervention with taxus and cardiac surgery score (SYNTAX) score (SS) was used to determine CAD severity by scoring system. SS has been proved to predict clinical outcomes not only in acute coronary syndrome (ACS) but also in stable CAD [3–5]. Identifying relevant factors associated with high SS and close monitoring during and after hospitalization can improve the prognosis of CAD patients. Various plasma biomarkers have been proved to associate with CAD, but very few of them can provide valid information about the severity of CAD [6–8]. Therefore, more new biomarkers are needed to assess the severity of CAD.

Several lines of evidence showed that microRNAs (miRNAs) regulate signaling pathways involved in cell proliferation and differentiation, which plays an important role in the pathogenesis of atherosclerosis [9–11]. Plasma miRNAs could be considered as promising biomarkers for the diagnosis and prognosis of these diseases, especially for CAD [12, 13]. miR-208b and miR-499 are involved in cardiogenesis, and they are the main regulators of left ventricular remodeling and cardiac hypertrophy and involved in mediating the differentiation of cardioblasts to cardiomyocytes [14–16]. Additionally, studies have revealed that miR-208b is highly expressed during myocardial infarction (MI) [17]. Zhang et al. found that the expression of downregulated miR-499 increased PDCD4 expression and protected endothelial cells (ECs) from inflammatory damage during CAD by the nuclear factor-kappa B (NF-*κ*B)/tumor necrosis factor-alpha (TNF-*α*) signaling pathway [18].

Although the role of miR-208b and miR-499 in the blood vessels has been reported, the association between levels of circulating miR-208b and miR-499 and severity of CAD has not been studied yet. In the present study, we aimed to evaluate the relationship of plasma miR-208b and miR-499 levels with CAD severity.

## 2. Methods

### 2.1. Study Population

Between April and November 2016, 195 consecutive patients with CAD who underwent coronary angiography (CAG) in Liaocheng People's Hospital were enrolled in this study. Diagnostic criteria were referred to ACCF/AHA Guideline for the Management of ST-elevation Myocardial Infarction or Non-ST-Elevation Acute Coronary Syndromes [19, 20]. The inclusion criteria were patients with CAD aged from 35 to 85 years, and the chest pain lasting <24 hours. The exclusion criteria were patients with known inflammatory disease, valvular heart disease and received anticoagulant and patients who had significant hepatic dysfunction or renal failure, cancer, or malignancy and had diseases of hematological and immune system. After these exclusions, 195 patients were enrolled. According to hospital records, baseline characteristics and past medical history including hypertension, diabetes mellitus, and smoking status were collected. The SS was determined by two experienced cardiologists who were blinded to the laboratory and clinical data of patients. Patients were divided into three groups according to the SS levels as following: high SS > 32, 22 < intermediate SS ≤ 32, and low SS ≤ 22. The study protocol was approved by the Medical Ethics Committee of Liaocheng People's Hospital. All procedures were in accordance with principles of Helsinki Declaration, and all patients provided informed consent.

### 2.2. Sample Collection and Storage

After admission, blood collection was performed from study subjects prior to the CAG procedures. Blood samples were collected using ethylenediaminetetraacetic acid tubes. After centrifugation, samples were transferred to RNase/DNase-free tubes and stored at −80°C.

### 2.3. Plasma MicroRNA Isolation and Validation

Total RNA was extracted using TRIzol reagent (Invitrogen, USA), and PrimeScript™ RT Master Mix (Takara, Japan) was used for the reverse transcription reaction according to the manufacturer's instructions. Quantitative real-time polymerase chain reaction was conducted using SYBR^®^ PrimeScript™ miRNA RT-PCR Kit (Takara, Japan). Cycle threshold (Ct) values were normalized to cel-miR-39 using the formula 2^−(Ct[miR] − Ct[cel‐miR‐39])^ and the relative expression levels of miRs were analyzed by the 2^−ΔΔCt^ method.

### 2.4. Statistical Analysis

Statistical analysis was performed using SPSS 23.0 version software (IBM Corp.). Shapiro-Wilk test was used to verify whether continuous data was normally distribution. Normally distributed data was expressed as mean ± standard deviation, and nonnormal distribution was presented as median (quartile deviation). Categorical variables were presented as counts (percentage). One-way analysis of variance (ANOVA) or the Kruskal-Wallis *H* test was used for comparisons among three groups. Chi-squared test was used to compare the categorical data. To analyze the differences of miR-208b and miR-499 expression intergroup, Steel-Dwass multiple comparisons tests were used for nonparametric variables post hoc analysis. Spearman's correlation test was used to analyze the correlation of SS and miR-208b and miR-499. Independent factors for predicting high SS were calculated by univariate analysis; variables with *p* value of <0.05 in univariate analysis were included in multivariate logistic regression models. Meanwhile, to further explore the applicability of using circulating miR-208b and miR-499 in predicting high SS, we performed receiver operating characteristic (ROC) curve analyses. All analyses were two-sided; the *p* value of <0.05 was determined as statistical significant. Steel-Dwass test was performed with free software (MEPHAS) available at http://www.gen-info.osaka-u.ac.jp/testdocs/tomocom/.

## 3. Results

### 3.1. Patient Characteristics

The study including 195 CAD patients who underwent CAG and the basic characteristics of patients are shown in Table 1. There were no significant differences in the proportion of age, gender, smoking status, and diabetes mellitus in the 3 groups. Laboratory parameters showed the levels of creatinine (Cr), creatine kinase isoenzymes (CK-MB), and high sensitivity C-reactive protein (hs-CRP) were higher in higher SS group than in lower SS group, as well as the mortality rate during hospitalization.

### 3.2. Plasma Levels of miR-208b and miR-499 Were Positively Correlated with the Severity of CAD

Patients with higher SS had significantly higher miR-208b and miR-499 levels compared with those with lower SS (*p* < 0.05) (Figure 1 and Table 2). Meanwhile, plasma miR-208b and miR-499 levels were positively associated with SS (Spearman's *r* = 0.535 and *r* = 0.407, respectively; both *p* < 0.001) (Figure 2). These results that indicated the increased expression of plasma miR-208b and miR-499 is significantly associated with the severity of CAD.

### 3.3. miR-208b and miR-499 Were Independent Predictors of the Severity of CAD

Multivariate logistic regression analysis was used to reveal the independent predictors of high SS using variables that showed statistically significant association in the univariate analysis. The result showed that miR-208b (odds ratio [OR]: 2.069; 95% confidence interval [CI]: 1.351-3.167; *p* = 0.001) and miR-499 (OR: 1.652; 95% CI: 1.222-2.233; *p* = 0.001) were independent predictors of high SS (Table 3).

### 3.4. Performance of miR-208b and miR-499 in the Prediction of Severity of CAD

To evaluate the performance of miR-208b and miR-499 in the prediction of high SS, ROC curves were performed (Figure 3). The area under the curve (AUC) values were 0.775 (*p* < 0.001) for miR-208b with 59% sensitivity and 88% specificity and the optimal cutoff value was 3.95; 0.713 (*p* < 0.001) for miR-499 with 54% sensitivity and 91% specificity and the optimal cutoff value was 5.19 in predicting high SS.

## 4. Discussion

According to our findings, we found that increased levels of miR-208b and miR-499 were significantly associated with CAD severity. All we know, this is the first study to report that miR-208b and miR-499 levels are independent predictors of high SS.

SS is usually used for calculating the severity and complexity of CAD and as a guideline for interventional cardiologist to choose more appropriate treatment between percutaneous coronary intervention (PCI) and coronary artery bypass graft surgery [21]. There is increasing evidence that has proven that this scoring system could predict major adverse cardiovascular events in patients with ACS or undergoing PCI [22, 23]. As in line with previous studies, in the present study, patients with higher SS have higher in-hospital mortality rate than patients with lower SS [7]. One of fundamental characteristics of atherogenesis is chronic inflammation and C-reactive protein (CRP) can reflect the inflammatory status. Previous study has demonstrated a close relationship between SS and inflammation [24]. Karadeniz and colleagues showed that hs-CRP level is associated with intermediate and high SS in patients with ACS [25]. In accordance with these findings, we observed that hs-CRP levels were significantly elevated in higher SS values and hs-CRP was an independent predictor of high SS. The identification of factors correlated with high SS may improve the prognosis of CAD patients. In our study, elevated CK-MB and leukocyte were also independent predictors of high SS. The relationship between CK-MB, leukocyte, and CAD severity has been established in previous studies [26, 27]. However, up to date, no study has investigated the association between miR-208b and miR-499 and severity of CAD. Our study indicated that miR-208b and miR-499 might be novel biomarkers for the severity of CAD.

Some pathological changes, including dysfunction of VSMCs and ECs, contribute to the formation of atherosclerosis [28]. VSMCs play a pivotal role in early progression of atherogenesis, which are the first cells present in atherosclerotic plaques. They secrete extracellular matrix that traps lipid from the bloodstream and can take up this lipid to form foam-like cells [29]. Arterial wall EC dysfunction could provoke monocyte adhesion initially, then followed by macrophage intruding the subendothelial area to form foam cells [28]. Circulating miR-208 is a cardiac-rich miRNA, presenting in two isoforms: miR-208a and miR-208b [30]. Zhang et al. [31] reported that miR-208 promotes VSMC proliferation via downregulation of its potential target-p21; in contrast, inhibition of miR-208 can reduce the effect on VSMC proliferation. Paradoxically, Zhou and coworkers found that miR-208b is highly expressed during MI and exerts its myocardioprotective effect against hypoxia-induced apoptosis, which can reduce EC apoptosis and attenuate atherosclerosis development [17, 32]. Further studies should be carried out to promote the understanding of the miR-208b functions in atherosclerosis. Recent study has shown that the expression of downregulated miR-499 increased PDCD4 expression and protected ECs from inflammatory damage during CAD through the NF-*κ*B/TNF-*α* signaling pathway [18]. Moreover, miR-499 overexpression suppressed its target gene—calcineurin A, which could induce EC inflammation and dysfunction [33, 34]. In our study, we observed that increased levels of miR-208b and miR-499 were significantly associated with higher SS, indicating that the two miRNAs could be potential targets for the treatment of CAD. Certainly, further studies that directly indicate the association of miR-208b and miR-499 and severity of CAD are warranted.

There may be several limitations in our study. First, it is a single-center study which involved a small sample size, and therefore; the predictive value of this study should be interpreted with caution. Second, in our study, we did not elucidate the mechanisms behind the association between circulating levels of miR-208b and miR-499 and severity of CAD. Therefore, larger clinical studies and some biological researches are required.

Overall, circulating miR-208b and miR-499 levels are significantly higher in higher SS patients compared to those in lower SS patients. miR-208b and miR-499 were found to be independent predictors of high SS. Our study may provide further evidence in the prediction of CAD severity for clinical implications.

## Figures and Tables

**Figure 1:** Relative expression of miR-208b (a) and miR-499 (b) in three groups. Abbreviation: SS: synergy between percutaneous coronary intervention with taxus and cardiac surgery (SYNTAX) score.

**Figure 2:** Correlation graph of miR-208b (a) and miR-499 (b) with SYNTAX score. Abbreviation: SYNTAX: synergy between percutaneous coronary intervention with taxus and cardiac surgery.

**Figure 3:** The receiver operating characteristic (ROC) curves of miR-208b (a) and miR-499 (b) in the prediction of high SYNTAX score. Abbreviation: SYNTAX: synergy between percutaneous coronary intervention with taxus and cardiac surgery; AUC: area under the curve; CI: confidence interval.

**Table 1:** Characteristics of patients according to SYNTAX score level.

	SS ≤ 22 (*n* = 43)	22 < SS ≤ 32 (*n* = 72)	SS > 32 (*n* = 80)	*p* value
Age (year)	60.19 ± 11.21	63.29 ± 10.25	64.58 ± 9.95	0.082
Male gender, *n* (%)	28 (65.12)	41 (56.94)	49 (61.25)	0.676
Smoking, *n* (%)	12 (27.91)	23 (31.94)	37 (46.25)	0.072
Hypertension, *n* (%)	19 (44.19)	51 (70.83)	51 (63.75)	0.016
DM, *n* (%)	5 (11.63)	15 (20.83)	23 (28.75)	0.088
Heart rate (bpm)	72.00 (12.00)	74.86 ± 11.46	78.00 (19.75)	0.025
Hemoglobin (g/L)	136.28 ± 14.91	137.56 ± 16.08	133.71 ± 14.10	0.281
Leukocyte (×10^9^/dL)	6.09 ± 1.58	6.17 ± 1.45	7.24 (2.56)	<0.001
Creatinine (*μ*mol/L)	65.79 ± 12.84	70.15 ± 17.68	67.79 ± 13.97	0.036
HDL (mmol/L)	1.28 (0.36)	1.25 (0.35)	1.23 ± 0.25	0.031
LDL (mmol/L)	2.66 ± 0.48	2.69 ± 0.74	2.59 ± 0.71	0.621
TC (mmol/L)	4.80 ± 1.05	4.64 (1.83)	4.52 (1.18)	0.742
CK-MB (IU/L)	11.51 ± 7.24	10.00 (4.75)	17.50 (16.50)	<0.001
Hs-CRP (mg/L)	1.04 (1.98)	0.88 (3.04)	3.84 (13.94)	<0.001
SS	12.00 (15.00)	27.00 (5.00)	43.5 (12.00)	<0.001
In-hospital mortality, *n* (%)	2 (4.65)	2 (2.78)	11 (13.75)	0.028

Abbreviation: SYNTAX: synergy between percutaneous coronary intervention with taxus and cardiac surgery; SS: SYNTAX score; DM: diabetes mellitus; HDL: high-density lipoprotein; LDL: low-density lipoprotein; TC: total cholesterol; CK-MB: creatine kinase isoenzyme; Hs-CRP: high-sensitivity C-reactive protein.

**Table 2:** Expression levels of circulating miRNA-208b and miRNA-499 in studied patients.

Variables	SS ≤ 22	22 < SS ≤ 32	SS > 32
	*n* = 43	*n* = 72	*n* = 80
miRNA-208b	1.78 (1.62)	3.32 ± 0.84^∗^	4..25±1.33^∗∗∗^
miRNA-499	2.43 (2.44)	4.52 (1.48)^∗^	5.42 (2.99)^∗∗∗^

^∗^ *p* < 0.05 when compared to 22 < SS ≤ 32 or SS > 32 with SS ≤ 22. ^∗∗^*p* < 0.05 when compared to 22 < SS ≤ 32 with SS > 32. Abbreviation: SS: synergy between percutaneous coronary intervention with taxus and cardiac surgery score.

**Table 3:** Logistic regression analysis for determining the independent predictors of high SS.

Variables	OR	95% CI	*p* value	Adjusted OR	95% CI	*p* value
Male gender	0.949	0.529-1.702	0.861			
Age	1.023	0.995-1.052	0.109			
Hypertension	1.113	0.627-2.039	0.684			
Diabetes mellitus	1.917	0.968-3.796	0.062			
Current smoking	1.967	1.088-3.557	0.025	2.019	0.805-5.064	0.134
Heart rate	1.036	1.013-1.060	0.002	1.031	0.994-1.069	0.099
Hemoglobin	0.985	0.968-1.004	0.126			
Leukocyte	1.472	1.230-1.761	<0.001	1.355	1.051-1.747	0.019
Hs-CRP	1.045	1.017-1.074	0.001	1.043	1.003-1.085	0.035
Creatinine	0.997	0.978-1.016	0.743			
CK-MB	1.125	1.067-1.185	<0.001	1.129	1.054-1.209	0.001
LDL-cholesterol	0.814	0.530-1.251	0.349			
HDL-cholesterol	0.215	0.069-0.664	0.008	0.336	0.060-1.884	0.215
Total cholesterol	0.987	0.774-1.259	0.919			
miRNA-208b	2.553	1.863-3.499	<0.001	2.069	1.351-3.167	0.001
miRNA-499	1.644	1.347-2.008	<0.001	1.652	1.222-2.233	0.001

Abbreviation: SS: synergy between percutaneous coronary intervention with taxus and cardiac surgery score; OR: odds ratio; CI: confidence interval; Hs-CRP: high-sensitivity C-reactive protein; CK-MB: creatine kinase isoenzyme; LDL: low-density lipoprotein; HDL: high-density lipoprotein.

## Data Availability

The data used to support the findings of this study are available from the corresponding author upon request.
